The article "Revealing the Effects of Corporate Governance on Green Investment and Innovation: Do Law and Policy Matter?" was retracted in 2025. Reasons: an official misconduct investigation; compromised peer review; a compromised editor; unreliable results or conclusions.

# Revealing the Effects of Corporate Governance on Green Investment and Innovation: Do Law and Policy Matter?

**DOI:** 10.3389/fpsyg.2022.961122

**Published:** 2022-07-19

**Authors:** Yuan Lai, Muhammad Tayyab Sohail

**Affiliations:** ^1^Faculty of Law, Macau University of Science and Technology, Taipa, Macao SAR, China; ^2^School of Public Administration, Xiangtan University, Xiangtan, China

**Keywords:** corporate governance, environmental law and policy, green investment and innovation, policy, sustainable

## Abstract

Green investment (GI) and innovation performance are key factors of sustainable green development. GI and innovation have become a trendy solution to minimize environmental issues in the previous few decades. We investigate the effects of corporate governance, environmental law, and environmental policy stringency on GI and environmental innovation (EI) using Chinese time-series data from 1998 to 2020. Short and long-run findings indicate that corporate governance has a positive and significant impact on GI and innovation in China. However, environmental law has positive and significant effects on GI and innovation in the short run and long run. Furthermore, environmental policy stringency has an insignificant impact on GI but stimulates green innovation both in the short and long run. The study also reveals that education has a significant positive impact on green innovation both in the short and long-run. The short and long-run results propose essential policy implications.

## Introduction

In recent times, global climate change has emerged as the most daunting challenge that humanity is facing. Even though implementation of the environmental regulations has helped to abate the environment-related issues up to some extent, they have also increased the economic costs of products and services. These deliberations inspire policymakers and empirics to look into the relationship between environmental laws, industry competitiveness, and the firms’ social duties (Greenstone et al., 2012; Kitzmueller and Shimshack, 2012; Arif and Sohail, 2020; Chai et al., 2021; Liu N. et al., 2022). In this regard, the researchers have focused on the various determinants of environmental efficiencies, such as public policies, energy policies, and technological innovations (Johnstone et al., 2010; Amores-Salvadó et al., 2014; Jian et al., 2021; Jiang et al., 2021); however, there are still a lot of variations inside the firms that can affect the environment and its related factors, which need further exploration. To fill this, lacuna researchers have recently started to explore the role of organizational structures in improving environmental efficiency (e.g., Martin et al., 2012; Sohail et al., 2013; Lin and Ho, 2016; Liu Y. et al., 2022). Several research works are available, confirming the positive role of management and organizational structures on environmental efficiency (Martin et al., 2012; Paillé et al., 2014; Sohail et al., 2014a,b). However, the direction of a causal relationship between the governance system and environmental quality is yet to be estimated in detail (Van Kamp et al., 2003; Khan et al., 2019, 2021a,b,2022a,b; Sohail et al., 2019a,b; Zhang et al., 2022; Zhenyu and Sohail, 2022).

Since the industrial revolution, most nations have adopted the process of industrialization but they have paid the environmental cost as well. Once the volume of industrialization increases, people become more and more aware of the environment-related issues (Ullah et al., 2020; Lu and Sohail, 2022; Sohail et al., 2022a,c, 2021d). Similarly, along with increasing environmental concerns, the firms started to focus more on improving their environmental efficiency (Wei et al., 2022). Therefore, the pressure is mounted on the firms and enterprises from all corners of the society, particularly, civil society, and environmentalists, to fulfill their responsibilities concerning environmental safety and protection. In this way, corporate social responsibility has gained popularity and has become a norm for modern enterprises to do business in recent times (Bénabou and Tirole, 2010; Shahab et al., 2016; Yasara et al., 2019; Sohail et al., 2021a,b,c,d; Khan et al., 2022a,b). In other words, the environmentally friendly conduct of the firms has got popularity as a helping hand in achieving sustainable development of the firms (Khan et al., 2021a,b). On one side, external factors are crucial in shedding light on the firm’s corporate responsibility regarding environmental sustainability (Leonidou et al., 2013; Yen et al., 2017, 2021; Yat et al., 2018; Zhao et al., 2019, 2022a,b; Sohail et al., 2020; Zahid et al., 2022). On the other side, several internal factors (e.g., competitive advantage, executive compensation, and corporate governance) are also important in explaining the firms’ environment-related policies (Muhammad et al., 2014: Mahfooz et al., 2017, 2019, 2020; Ji et al., 2021).

Currently, theorists and empirics have not reached any consensus on the matters related to environmental and green investment (GI). In this context, two different opinions have come to the fore. According to traditional opinion, green or environmental investment is purely a cost (Schaltegger and Synnestvedt, 2002); in contrast, the modern view suggests that environmental investment can bring future prosperity (Porter and Van der Linde, 1995; Sánchez-Medina et al., 2015; Jiang and Akbar, 2018). In recent times, GI has become part and parcel of the firm’s environmental strategy. Given the importance of the GI by firms in protecting the environment, various factors have been recorded as a promoter of GI, including green fees, eco-innovation, environmental technologies, waste discharge fees, pollution penalties, and so on. Increasing the number of green investors may positively impact the firm’s environmental strategy and social responsibility (Chuang and Huang, 2018). Clement and Meunie (2010) analyzed the role of social responsibility, GI, and cultural norms played in improving environmental quality. According to Chuang and Huang (2018), corporate social responsibility exerted a positive impact on green information technology, green communication capital structure, and green capital linkage. Moreover, they observed that green capital help improve environmental performance, which consequently improves business competition. Similarly, Guenster et al. (2011) also observed a positive relationship between a firm’s environmental performance and its corporate worth.

Another important relationship that has recently come in limelight is the link between corporate governance and green innovation. Certainly, modern-day firms have become more serious about investing in green research and development activities that would lead them toward the path of eco-innovations (Khan et al., 2020a,b; Chen et al., 2022; Li et al., 2022a,b,c). However, going green is relatively a newer concept that requires a shift in the firm’s research and development culture, the introduction of new production techniques, investment in green technologies, and promotion of novel ideas (Sohail et al., 2014b; Rasool et al., 2017; Khan et al., 2018a,b; Usman et al., 2021; Li and Ullah, 2022; Mustafa et al., 2022). Therefore, Kock et al. (2012) observed that “successfully reducing and preventing waste emissions necessitates a great deal of extra managerial effort because it requires a complex redesign of a firm’s internal processes and the development of green competencies.” The Organization of Economic Cooperation and Development (OECD) underlined that the conventional business model adopted by the traditional firms stops them from being involved in a more radical method of eco-innovation. According to OECD, many existing firms are more than satisfied with their existing business model and do not involve in systematic efforts to bring more radical technological innovations. Therefore, more complex research and development questions are to be answered if the firms want to involve technological innovations. However, it is widely accepted that managerial entrenchment is a hurdle in the way of managerial inclinations toward complex activities; hence, we can confer that worse corporate governance is negatively related to green innovation.

While the environmental benefits are widely considered to be the by-product of environment-related regulations (Magazzino and Falcone, 2022), the debate among the empirics on this topic is still on. The available literature in this regard suggests that firms and industries have to bear the extra cost due to the implementation of strict rules and regulations that may negatively impact the firms’ competitive position, profitability, production, demand, and investment decisions (Kozluk and Zipperer, 2015; Sohail et al., 2015). However, a modern view of the relationship between environmental aims and firms’ benefits may go side by side with each other, and law and regulation may serve as a “win-win” situation for the firm because it can increase its long-term profitability and improve competitive position (Porter and Van der Linde, 1995). Previously, empirics have tried to find the various factors that affect green investment and innovation, but none have focused on the impact of corporate governance on green investment and innovation in China’s economy. This study will fill this gap in the literature and analyze the impact of corporate governance on green investment and innovation in China’s economy, which is the first of its kind. This study will try to answer the following research questions: (1) does corporate governance lead to promote green investment and innovation? (2) Do environmental law and policy matter for green investment and innovation?

This new perspective has given rise to a new debate under the porter hypothesis; the main focus of which is to observe the link between related laws and regulations and innovations. This linkage is considered an important element in improving a firm’s performance. Keep in mind that with the above discussion, we aim to investigate the impact of corporate governance, environmental law, and environmental policy stringency on green investment and innovation in China by using the ARDL method. This technique works better on a small sample and provides relatively more robust results. This approach also provides short and long-run effects of corporate governance, environmental law, and environmental policy stringency on green investment and innovation.

## Empirical Methods

The main aim of this paper is to identify the effect of corporate governance, environmental law, and environmental policy stringency on green investment and innovation, using the China data over the period 1998–2020. Our empirical model is based on stakeholder–agency theory and porter’s innovation theory (Porter, 1991; Hill and Jones, 1992). Theoretically, standard green investment and innovation are associated with corporate governance, environmental law, and environmental policy stringency. Therefore, standard time series models will be:


$${\text{EI}}_{\text{t}}=\pi_{0}+\pi_{1}\,{\text{BI}}_{\text{t}}+\pi_{2}\,{\text{ER}}_{\text{t}}+\pi_{3}\,{\text{EPS}}_{\text{t}}$$

(1) $$\;\;+\pi_{4}\,{\text{Education}}_{\text{t}}+\varepsilon_{\text{t}}$$

$${\text{GI}}_{\text{t}}=\pi_{0}+\pi_{1}\,{\text{BI}}_{\text{t}}+\pi_{2}\,{\text{ER}}_{\text{t}}+\pi_{3}\,{\text{EPS}}_{\text{t}}$$

(2) $$\;\;+\pi_{4}\,{\text{Education}}_{\text{t}}+\varepsilon_{\text{t}}$$

Where the dependent variables are the EI and GI that are assumed to depend on the corporate governance (CG), environmental regulations (ER), environmental policy stringency (EPS), and educational attainment (Education). Equations (1) and (2) are long-run models and estimates of π_1_, π_2_,  π_3_, and π_4_ reflect long-run effects of variables corporate governance, environmental law, environmental policy stringency, and education on EI and GI. To assess the short-run effects, we need to re-write Equations (1) and (2) in an error-correction format so that we can also judge the short-term effects of corporate governance, environmental law, environmental policy stringency, and education. A method that offers long-term and short-term estimates in one step is that of Pesaran et al. (2001) ARDL bounds testing approach. In doing so, we follow the ARDL method and rely on the following error-correction specification:


$$\Delta \,{\mathrm{EI}}_{\text{t}}=\pi_{0}+\,\sum_{\text{k}=1}^{\text{n}}\beta_{1\,\text{k}}\,\Delta \,{\mathrm{EI}}_{t-\text{k}}+\,\sum_{\text{k}=0}^{\text{n}}\beta_{2\,\text{k}}\,\Delta \,{\mathrm{BI}}_{\text{t}-\text{k}}$$

$$\;\;+\sum_{\text{k}=1}^{\text{n}}\beta_{3\,\text{k}}\,\Delta \,{\mathrm{ER}}_{t-\text{k}}+\,\sum_{\text{k}=0}^{\text{n}}\beta_{4\,\text{k}}\,\Delta \,{\mathrm{EPS}}_{\text{t}-\text{k}}$$

$$\;\;+\sum_{\text{k}=1}^{\text{n}}\beta_{5\,\text{k}}\,\Delta \,{\mathrm{Education}}_{t-\text{k}}+\pi_{1}\,{\text{EI}}_{\text{t}-1}+\pi_{2}\,{\text{BI}}_{\text{t}-1}$$

$$\;\;+\pi_{3}\,{\text{ER}}_{\text{t}-1}+\pi_{4}\,{\text{EPS}}_{\text{t}-1}+\pi_{5}\,{\text{Education}}_{\text{t}-1}$$

(3) $$\;\;+\lambda .{\mathrm{ECM}}_{\text{t}-1}+\varepsilon_{\text{t}}$$

$$\Delta \,{\mathrm{GI}}_{\text{t}}=\pi_{0}+\,\sum_{\text{k}=1}^{\text{n}}\beta_{1\,\text{k}}\,\Delta \,{\mathrm{GI}}_{t-\text{k}}+\,\sum_{\text{k}=0}^{\text{n}}\beta_{2\,\text{k}}\,\Delta \,{\mathrm{BI}}_{\text{t}-\text{k}}$$

$$\;\;+\sum_{\text{k}=1}^{\text{n}}\beta_{3\,\text{k}}\,\Delta \,{\mathrm{ER}}_{t-\text{k}}+\,\sum_{\text{k}=0}^{\text{n}}\beta_{4\,\text{k}}\,\Delta \,{\mathrm{EPS}}_{\text{t}-\text{k}}$$

$$\;\;+\sum_{\text{k}=1}^{\text{n}}\beta_{5\,\text{k}}\,\Delta \,{\mathrm{Education}}_{t-\text{k}}+\pi_{1}\,{\text{GI}}_{\text{t}-1}+\pi_{2}\,{\text{BI}}_{\text{t}-1}$$

$$\;\;+\pi_{3}\,{\text{ER}}_{\text{t}-1}+\pi_{4}\,{\text{EPS}}_{\text{t}-1}+\pi_{5}\,{\text{Education}}_{\text{t}-1}$$

(4) $$\;\;+\lambda .{\mathrm{ECM}}_{\text{t}-1}+\varepsilon_{\text{t}}$$

In both Equations (3) and (4), the coefficients assigned to the “B” are short-run effects and the estimates of π_1_ – π_5_ are the long-run effects. Standard literature proposes two tests for establishing cointegration among the variables, such as *F*-test and *t*-test. Previous other co-integration methods do not offer robust estimates and have some limitations. ARDL approach cannot be used when variables are not stationary, as this approach needs all the series to be integrated of either I (0) or I (1), or contains a mixture of the order of integration (Bahmani-Oskooee et al., 2020). The level of integration has been determined by using PP and DF-GLS unit root tests (Zhou et al., 2022). This technique becomes more suitable for limited sample data, as in the case of China. This method directly explores short-run, as well long-run effects, in a single step. This method offers correct estimations of the long-term model. Moreover, ARDL is free from residual correlation and endogeneity. Serial correlation is verified through the Lagrange multiplier (LM). The model specification is checked using the Ramsey RESET test. This study employs the CUSUM and CUSUM-sq tests to check the model stability.

### Data

This study examines the effect of corporate governance, law, and policy on green investment and innovation. Table 1 provides information about abbreviations and definitions of variables and their source of data. Table 2 reported descriptive statistics. In this study, green investment is measured through nuclear, renewables, and others in terms of quad Btu, and the data has been taken from EIA. Environment-related technologies data has been explored by OECD. Board independence is used to measure corporate governance which refers to the proportion of independent directors to the total number of directors on a board. The data for board independence is taken from China’s stock market and accounting research. Environmental regulations (measured as environment-related taxes as a percent of total tax revenue) have been used to measure environmental law impact. While environmental policy stringency is used to measure policy impact. The data for environmental regulation and environmental policy stringency is taken from the OECD. Education measured as average years of schooling has been added as a control variable and the data is extracted from the study of Barro and Lee.

**TABLE 1:** Definitions and data sources.

Variables	Abbreviations	Definitions	Data sources
Green investment	GI	Nuclear, renewables, and other (quad Btu)	EIA
Environmental innovation	EI	Environment-related-technologies	OECD
Board independence	BI	Board Independence refers to the proportion of independent directors to the total number of directors on board.	CSMAR
Environmental regulation	ER	Environmentally related taxes, % total tax revenue	OECD
Environmental policy stringency	EPS	Environmental policy stringency index ranges from 0 (not stringent) to 6 (highest degree of stringency)	OECD
Year of schooling	Education	Average year of schooling	Barro and Lee

**TABLE 2:** Descriptive statistics.

	Mean	Median	Maximum	Minimum	Std. dev.	Skewness	Kurtosis
GI	9.325	7.157	22.24	2.226	6.578	0.661	2.090
EI	10.35	10.43	12.28	8.210	1.284	–0.175	1.791
BI	0.403	0.360	0.764	0.010	0.227	–0.323	2.246
ER	3.671	3.100	6.360	1.564	1.498	0.411	1.790
EPS	1.257	0.980	2.210	0.520	0.632	0.281	1.407
Education	12.16	12.60	14.65	9.300	1.830	–0.275	1.610

## Results and Discussion

Our study is based on time-series data and the prerequisite of applying the regression technique is to confirm the stationarity of variables to be used in the model. Thus, two-unit root tests have been chosen for this exercise. Table 3 reports the results of the PP unit root test and DF-GLS unit root test. Both tests report similar order of integration. It displays that only education is at stationary level, while, GI, EI, BI, ER, and EPS are stationary at first difference. Hence, the precondition to applying the ARDL approach, i.e., the mixed order of integration, is fulfilled. Table 4 is reporting the result estimates of green investment and EI models. The upper panel provides the short-run estimates of both models, the middle panel contains long-run estimates, and the lower panel reports the findings of some important diagnostic tests.

**TABLE 3:** Unit root testing.

	PP		DF-GLS			
		
	I (0)	I (1)	I (0)	I (1)	PP	DF-GLS
GI	1.754	–2.987*	–1.234	–1.814*	I(1)	I (1)
EI	–1.03	–2.875*	0.123	–4.302***	I(1)	I (1)
BI	–0.754	–3.120**	–0.542	–3.012***	I(1)	I (1)
ER	–1.023	–3.012**	–0.875	–3.012***	I(1)	I (1)
EPS	–0.421	–3.874***	–0.185	-3.012***	I(1)	I (1)
Education	–2.675*		–1.675*		I(0)	I (0)

***p < 0.01; **p < 0.05; *p < 0.1.

**TABLE 4:** Estimates of green investment and environmental innovation.

	Green investment				Environmental innovation			
		
Variable	Coefficient	Std. error	t-statistic	Prob.*	Coefficient	Std. error	*t*-statistic	Prob.*
**Short-run**								
BI	2.904***	0.827	3.512	0.177	3.216***	0.203	15.85	0.040
BI (–1)	2.584***	0.735	3.514	0.177	1.358***	0.174	7.796	0.081
BI (–2)	0.045	0.127	0.357	0.782	1.933***	0.204	9.466	0.067
ER	0.425***	0.091	4.684	0.134	0.030***	0.006	4.888	0.129
ER (–1)	1.388***	0.100	13.88	0.046	0.008	0.015	0.508	0.701
ER (–2)	0.621***	0.231	2.692	0.226	0.074***	0.016	4.636	0.135
EPS	0.196	0.290	0.676	0.622	0.082***	0.028	2.964	0.207
EPS (–1)	0.479*	0.274	1.750	0.331	0.377***	0.036	10.56	0.060
EPS (–2)	–5.215***	0.387	–13.46	0.047	–0.305***	0.064	–4.757	0.132
EPS (–3)	0.537	0.567	0.946	0.518	0.245***	0.039	6.342	0.100
EDUCATION	3.122***	0.447	6.983	0.091	0.142**	0.058	2.439	0.248
EDUCATION (–1)	3.398***	0.410	8.295	0.076	0.056	0.046	1.199	0.443
EDUCATION (–2)	–1.712***	0.332	–5.155	0.122	0.077	0.052	1.484	0.378
**Long-run**								
BI	2.533***	10.43	0.243	0.812	2.294***	0.063	36.22	0.018
ER	2.730***	0.796	3.428	0.004	0.009***	0.003	3.477	0.178
EPS	0.854	3.040	0.281	0.783	0.184***	0.018	10.05	0.063
EDUCATION	6.834***	2.591	2.638	0.020	0.478***	0.005	98.14	0.007
C	11.37***	0.871	13.05	0.004	4.137***	0.054	76.26	0.008
**Diagnostics**								
*F*-test	8.021***				14.02***			
ECM (–1)*	–0.725***	0.007	–98.24	0.007	–0.409***	0.138	–2.972	0.010
LM	2.012				1.065			
RESET	1.032				0.701			
CUSUM	S				S			
CUSUM	S				S			

***p < 0.01; **p < 0.05; *p < 0.1.

The long-run findings show that board independence is significantly and positively associated with green investment and EI displaying that corporate governance tends to enhance green investment and EI in the case of China. It infers that a 1% upsurge in board independence increases green investment by 2.533% and EI by 2.294% in the long run. This finding is supported by Hill and Jones (1992) stakeholder–agency theory, which noted that corporate governance increases return on shareholder green investment by minimizing pollution levels. This theory provides a positive effect of corporate governance on environmental performance. This finding also infers that green innovation and investment are executive’s strategic decisions. This finding is also in line with Abebe and Myint (2018), who noted that the board of directors encourages companies to adopt an innovation-based green business model. This means that the board of directors cannot separate the economic objectives from the environmental issues. Therefore, companies increase profits in an ethical and environmentally responsible manner to meet the interests of the green economy. A similar finding is also suggested by previous studies (see Amore and Bennedsen, 2016; Asni and Agustia, 2022). This means that corporate governance is an essential organ in green development by encouraging green investment and innovation.

Environmental regulation is also significantly and positively linked with green investment and EI in the long run, demonstrating that implementation of environmental law tends to improve green investment and EI in the case of China. It concludes that a 1% upsurge in implementation of environmental regulation increases green investment by 2.730% and EI by 0.009% in the long run. This finding is backed by Porter’s Hypothesis (Porter, 1991), which noted that stricter environmental regulation fosters green innovation, which in turn increases green productivity and firm’s competitiveness. This means that environmental laws and regulations enforce firms for green investment and innovation. This also infers that environmental laws and regulations trigger society and firms for dynamic green efficiency. This finding is also backed by Huang and Lei (2021), who suggest that environmental regulation is positively related to green investment in China due to legal requirements.

Environmental policy stringency is significantly and positively attached to EI confirming that environmental policy stringency tends to enhance EI in China in the long-run. It infers that a 1% upsurge in environmental policy stringency enhances EI by 0.184% in the long run. In contrast, the association between environmental policy stringency and green investment is found insignificant in the long run, revealing no impact of environmental policy on green investment in China hereafter. This finding is also empirically supported by Hassan and Rousselière (2022), who suggested that strict environmental policy leads to enhanced green innovation in OECD. Education is significantly and positively associated with green investment and EI, in the long run, inferring that education tends to improve green investment and EI in China. It reveals that a 1% increase in education increases green investment by 6.834% and EI by 0.478% in due course.

In the short run, findings infer that board independence is significantly and positively associated with green investment and EI confirming that corporate governance also contributes significantly to the improvement of green investment and EI in the short term. It reveals that a 1% upsurge in board independence increases green investment by 2.904% and environmental innovation by 3.216% in the long run. Environmental regulation also reports a significant and positive impact on green investment and EI in the short run, showing that implementation of environmental regulations improves green investment and EI in case of China. It concludes that a 1% rise in environmental regulation increases green investment by 0.425% and EI by 0.030% in the short run. Environmental policy stringency is significantly and positively associated with EI, confirming that environmental policy stringency tends to enhance EI in the short run. It infers that 1% rise in environmental policy stringency enhances EI by 0.082% in the short run as well. In contrast, the nexus between environmental policy stringency and green investment is found insignificant in the short run. Education is significantly and positively associated with green investment and EI in the short run, inferring that education tends to improve green investment and EI in the case of China. It reveals that a 1% increase in education increases green investment by 3.122% and EI by 0.142% in the long-run.

The diagnostic tests are performed to validate the findings of ARDL models. The findings of all diagnostics tests are according to our expectations. The findings of the *F*-test and ECM tests validate the long-run cointegration relationship among variables. LM test reveals that no issue of serial correlation is found in both models. Model specification is confirmed through the results of the Ramsey RESET test. The stability of the results is confirmed by the findings of CUSUM tests in Table 4 and Figures 1, 2.

**FIGURE 1:** Plots of CUSUM and CUSUM-sq (green investment).

**FIGURE 2:** Plots of CUSUM and CUSUM-sq (environmental innovation).

## Conclusion and Implications

It is essential to encourage green investment and innovation through corporate governance, effectively formulating environmental regulations and environmental policies that stimulate green investment and innovation. Thus, this study intends to explore the impact of corporate governance, environmental regulation, and environmental policy stringency on green investment and innovation. In this study, corporate governance is measured by board independence. Environmental law is measured through environmental regulations, while the environmental policy is measured through environmental stringency policy. Education role has been included as a control variable. For deducing long-run and short-run estimates, the study adopted the ARDL approach and reported the following findings. Firstly, the long-run finding reveals that board independence reports a significant and positive effect on GI and EI, revealing that corporate governance can be adopted as a policy tool to enhance GI and EI in China. Secondly, environmental regulations also show a positive association with GI and EI, confirming that implementation of environmental laws is necessary to enhance GI and EI in China. Thirdly, environmental policy stringency shows a positive association with EI, confirming that the effectiveness of environmental policies can contribute significantly to enhancing EI in China. Lastly, education is proven to be positively associated with GI and EI. Hence, this study concludes that corporate governance, environmental regulation, environmental policy stringency, and education are effective determinants of GI and EI.

Based on these findings, this research offers the following policy suggestions. Based on the positive impact of board independence on GI and eco-innovation, this study suggests that optimization of the mechanism of corporate governance as a policy tool to attain sustainability of the organization through GI and EI according to the expectations of the stakeholders. In this way, the organization can attain the competence of directors, skills, and experience to enhance the performance of EI and GI. There is a need to control the influence of large investors to enhance the implementation of GI and EI as these investors can significantly influence the decision-making powers of management. Additionally, environmental determinants should be involved in the performance measurement procedure of local governments. The findings of this study support policymakers and environmentalists to design more effective environmental laws. The Chinese government should adopt environmental regulations and environmental policy stringency in a manner that promotes the GI in the country and also stimulates the firms to invest more in the R and D sector to enhance EI.

Our study contains a few limitations that need to be considered in future studies. Our study considers only one direction of corporate governance; however, there are various measures of corporate governance, such as senior executive dynamic capabilities, environmental legitimacy, quality management, and market competition. Future studies should incorporate these measures into analysis to get a more accurate effect of corporate governance on innovation and GI. Future studies should make comparisons between developed and developing economies by replicating the objectives of this study. Future studies can also explore the impact of corporate governance on environmental sustainability and clean energy consumption.

## Data Availability Statement

The raw data supporting the conclusions of this article will be made available by the authors, without undue reservation.

## Author Contributions

YL gave this idea and read and approved the final version. YL and MS wrote the manuscript. Both authors contributed to the article and approved the submitted version.

## Conflict of Interest

The authors declare that the research was conducted in the absence of any commercial or financial relationships that could be construed as a potential conflict of interest.

## Publisher’s Note

All claims expressed in this article are solely those of the authors and do not necessarily represent those of their affiliated organizations, or those of the publisher, the editors and the reviewers. Any product that may be evaluated in this article, or claim that may be made by its manufacturer, is not guaranteed or endorsed by the publisher.

## References

[B1] AbebeM.MyintP. P. A. (2018). Board characteristics and the likelihood of business model innovation adoption: evidence from the smart home industry. *Int. J. Innovat. Manag.* 22:1850006. 10.1142/S1363919618500068

[B2] AmoreM. D.BennedsenM. (2016). Corporate governance and green innovation. *J. Environ. Econ. Manag.* 75 54–72. 10.1016/j.jeem.2015.11.003

[B3] Amores-SalvadóJ.Martín-de CastroG.Navas-LópezJ. E. (2014). Green corporate image: moderating the connection between environmental product innovation and firm performance. *J. Cleaner Product.* 83 356–365. 10.1016/j.jclepro.2014.07.059

[B4] ArifU.SohailM. T. (2020). Asset pricing with higher co-moments and CVaR: evidence from pakistan stock exchange. *Int. J. Econ. Financial Issues* 10:243. 10.32479/ijefi.10351

[B5] AsniN.AgustiaD. (2022). Does corporate governance induce green innovation? an emerging market evidence. *Corp. Governance: Int. J. Bus. Soc.* Online ahead of print

[B6] Bahmani-OskooeeM.UsmanA.UllahS. (2020). Asymmetric impact of exchange rate volatility on commodity trade between Pakistan and China. *Global Bus. Rev.* 1-25. 10.1177/0972150920916287

[B7] BénabouR.TiroleJ. (2010). Individual and corporate social responsibility. *Economica* 77 1–19. 10.1111/j.1468-0335.2009.00843.x

[B8] ChaiM.DengY.SohailM. T. (2021). “Study on synergistic mechanism of water environment governance in dongting lake basin based on evolutionary game,” in *Proceedings of the E3S Web of Conferences*, Vol. 257 (Les Ulis: EDP Sciences), 03075. 10.1051/e3sconf/202125703075

[B9] ChenJ.RojniruttikulN.KunL. Y.UllahS. (2022). Management of green economic infrastructure and environmental sustainability in one belt and road enitiative economies. *Environ. Sci. Pollut. Res.* 29 36326–36336. 10.1007/s11356-021-18054-5 35060037

[B10] ChuangS. P.HuangS. J. (2018). The effect of environmental corporate social responsibility on environmental performance and business competitiveness: the mediation of green information technology capital. *J. Bus. Ethics* 150 991–1009. 10.1007/s10551-016-3167-x

[B11] ClementM.MeunieA. (2010). Is inequality harmful for the environment? an empirical analysis applied to developing and transition countries. *Rev. Soc. Econ.* 68 413–445. 10.1080/00346760903480590 21280382

[B12] GreenstoneM.ListJ. A.SyversonC. (2012). *The Effects of Environmental Regulation on the Competitiveness of US Manufacturing (No. w18392).* Cambridge, MA: National Bureau of Economic Research. 10.3386/w18392

[B13] GuensterN.BauerR.DerwallJ.KoedijkK. (2011). The economic value of corporate eco-efficiency. *Eur. Financial Manag.* 17 679–704. 10.1111/j.1468-036X.2009.00532.x

[B14] HassanM.RousselièreD. (2022). Does increasing environmental policy stringency lead to accelerated environmental innovation? a research note. *Appl. Econ.* 54 1989–1998. 10.1080/00036846.2021.1983146

[B15] HillC. W.JonesT. M. (1992). Stakeholder-agency theory. *J. Manage. Stud*. 29, 131–154.

[B16] HuangL.LeiZ. (2021). How environmental regulation affect corporate green investment: evidence from China. *J. Cleaner Product.* 279:123560. 10.1016/j.jclepro.2020.123560

[B17] JiX.ZhangY.MirzaN.UmarM.RizviS. K. A. (2021). The impact of carbon neutrality on the investment performance: evidence from the equity mutual funds in BRICS. *J. Environ. Manage.* 297:113228. 10.1016/j.jenvman.2021.113228 34273643

[B18] JianL.SohailM. T.UllahS.MajeedM. T. (2021). Examining the role of non-economic factors in energy consumption and CO2 emissions in China: policy options for the green economy. *Environ. Sci. Pollut. Res.* 28 67667–67676. 10.1007/s11356-021-15359-3 34263395

[B19] JiangA.CaoY.SohailM. T.MajeedM. T.SohailS. (2021). Management of green economy in China and India: dynamics of poverty and policy drivers. *Environ. Sci. Pollut. Res.* 28 55526–55534. 10.1007/s11356-021-14753-1 34138433

[B20] JiangX.AkbarA. (2018). Does increased representation of female executives improve corporate environmental investment? evidence from China. *Sustainability* 10:4750. 10.3390/su10124750

[B21] JohnstoneN.HaščičI.PoppD. (2010). Renewable energy policies and technological innovation: evidence based on patent counts. *Environ. Resource Econ.* 45 133–155. 10.1007/s10640-009-9309-1

[B22] KhanM. K.AliR.TariqS. (2018a). Impact of ownership structure on corporate dividend policy and performance. *KASBIT Bus. J.* 11 110–130.

[B23] KhanM. K.HeY.KaleemA.AkramU.HussainZ. (2018b). Remedial role of financial development in corporate investment amid financing constraints and agency costs. *J. Bus. Econ. Manag.* 19 176–191. 10.3846/16111699.2017.1422797

[B24] KhanM. K.AliS.ZahidR. A.HuoC.NazirM. S. (2022a). Does whipping tournament incentives spur CSR performance? an empirical evidence from chinese sub-national institutional contingencies. *Front. Psychol.* 13:841163. 10.3389/fpsyg.2022.841163 35282226PMC8913534

[B25] KhanM. K.NaeemK.HuoC.HussainZ. (2022b). The nexus between vegetation, urban air quality, and public health: an empirical study of lahore. *Front. Public Health* 10:842125. 10.3389/fpubh.2022.842125 35558537PMC9086906

[B26] KhanM. K.IqbalM. A.BratovV.MorozovN. F.GuptaN. K. (2020a). An investigation of the ballistic performance of independent ceramic target. *Thin-Walled Struct.* 154:106784. 10.1016/j.tws.2020.106784

[B27] KhanM. K.ZulfiqarS.HussainA. (2020b). Innovation and investment in high-tech firms in financially constrained environment. *Acad. J. Soc. Sci. (AJSS)* 4 187–207. 10.54692/ajss.2020.04021042

[B28] KhanM. K.KaleemA.ZulfiqarS.AkramU. (2019). Innovation investment: behaviour of Chinese firms towards financing sources. *Int. J. Innovat. Manag.* 23:1950070. 10.1142/S1363919619500701

[B29] KhanM. K.QinY.ZhangC. (2021a). Financial structure and earnings manipulation activities in China. *World Econo.* 1–31. 10.1111/twec.13232

[B30] KhanM. K.ZahidR. A.SaleemA.SágiJ. (2021b). Board composition and social & environmental accountability: a dynamic model analysis of Chinese firms. *Sustainability* 13:10662. 10.3390/su131910662

[B31] KitzmuellerM.ShimshackJ. (2012). Economic perspectives on corporate social responsibility. *J. Econ. Literature* 50 51–84. 10.1257/jel.50.1.51

[B32] KockC. J.SantalóJ.DiestreL. (2012). Corporate governance and the environment: what type of governance creates greener companies? *J. Manag. Stud.* 49 492–514. 10.1111/j.1467-6486.2010.00993.x

[B33] KozlukT.ZippererV. (2015). Environmental policies and productivity growth: a critical review of empirical findings. *OECD J. Econ. Stud.* 2014 155–185. 10.1787/eco_studies-2014-5jz2drqml75j

[B34] LeonidouC. N.KatsikeasC. S.MorganN. A. (2013). “Greening” the marketing mix: do firms do it and does it pay off? *J. Acad. Market. Sci.* 41 151–170. 10.1007/s11747-012-0317-2

[B35] LiW.UllahS. (2022). Research and development intensity and its influence on renewable energy consumption: evidence from selected Asian economies. *Environ. Sci. Pollution Res.* Online ahead of print. 10.1007/s11356-022-19650-9 35303227

[B36] LiX.ShaikhP. A.UllahS. (2022a). Exploring the potential role of higher education and ICT in China on green growth. *Environ. Sci. Pollution Res.* 10.1007/s11356-022-20292-0 35474423

[B37] LiY.ChenJ.SohailM. T. (2022b). Does education matter in China? myths about financial inclusion and energy consumption. *Environ. Sci. Pollution Res.* Online ahead of print. 10.1007/s11356-022-21011-5 35624362

[B38] LiY.ChenJ.SohailM. T. (2022c). Financial Inclusion and their Role in Renewable Energy and Non-renewable Energy Consumption in China: Exploring the Transmission Channels. *Res. Square* [Preprint] 1–15. 10.21203/rs.3.rs-1355688/v1

[B39] LinL. H.HoY. L. (2016). Institutional pressures and environmental performance in the global automotive industry: the mediating role of organizational ambidexterity. *Long Range Plann.* 49 764–775.

[B40] LiuN.HongC.SohailM. T. (2022). Does financial inclusion and education limit CO2 emissions in China? a new perspective. *Environ. Sci. Pollution Res.* 29 18452–18459. 10.1007/s11356-021-17032-1 34687414

[B41] LiuY.SohailM. T.KhanA.MajeedM. T. (2022). Environmental benefit of clean energy consumption: can BRICS economies achieve environmental sustainability through human capital? *Environ. Sci. Pollution Res.* 29 6766–6776. 10.1007/s11356-021-16167-5 34460087

[B42] LuF.SohailM. T. (2022). Exploring the effects of natural capital depletion and natural disasters on happiness and human wellbeing: a study in China. *Front. Psychol.* 13:870623. 10.3389/fpsyg.2022.870623 35677125PMC9168647

[B43] MagazzinoC.FalconeP. M. (2022). Assessing the relationship among waste generation, wealth, and GHG emissions in Switzerland: some policy proposals for the optimization of the municipal solid waste in a circular economy perspective. *J. Cleaner Product.* 351:131555. 10.1016/j.jclepro.2022.131555

[B44] MahfoozY.YasarA.GuijianL.YousafB.SohailM. T.KhanS. (2020). An assessment of wastewater pollution, treatment efficiency and management in a semi-arid urban area of Pakistan. *Desalination Water Treat* 177 167–175. 10.5004/dwt.2020.24949 26354686

[B45] MahfoozY.YasarA.SohailM. T.TabindaA. B.RasheedR.IrshadS. (2019). Investigating the drinking and surface water quality and associated health risks in a semi-arid multi-industrial metropolis (Faisalabad), Pakistan. *Environ. Sci. Pollution Res.* 26 20853–20865. 10.1007/s11356-019-05367-9 31111390

[B46] MahfoozY.YasarA.TabindaA. B.SohailM. T.SiddiquaA.MahmoodS. (2017). Quantification of the River Ravi pollution load and oxidation pond treatment to improve the drain water quality. *Desalin Water Treat* 85 132–137. 10.5004/dwt.2017.21195 26354686

[B47] MartinR.MuûlsM.De PreuxL. B.WagnerU. J. (2012). Anatomy of a paradox: management practices, organizational structure and energy efficiency. *J. Environ. Econ. Manag.* 63 208–223. 10.1016/j.jeem.2011.08.003

[B48] MuhammadA. M.ZhonghuaT.DawoodA. S.SohailM. T. (2014). A study to investigate and compare groundwater quality in adjacent areas of landfill sites in lahore city. *Nat. Environ. Pollution Technol.* 13 1–10.

[B49] MustafaS.SohailM. T.AlroobaeaR.RubaieeS.AnasA.OthmanA. M. (2022). Éclaircissement to understand consumers’ decision-making psyche and gender effects, a fuzzy set qualitative comparative analysis. *Front. Psychol*. 13:920594. 10.3389/fpsyg.2022.920594 35719580PMC9201776

[B50] PailléP.ChenY.BoiralO.JinJ. (2014). The impact of human resource management on environmental performance: an employee-level study. *J. Bus. Ethics* 121 451–466. 10.1007/s10551-013-1732-0

[B51] PesaranM. H.ShinY.SmithR. J. (2001). Bounds testing approaches to the analysis of level relationships. *J. Appl. Econ.* 16 289–326. 10.1002/jae.616

[B52] PorterM. (1991). America’s green strategy. *Sci. Am. Magazine* 264:168. 10.1038/scientificamerican0491-168

[B53] PorterM. E.Van der LindeC. (1995). Toward a new conception of the environment-competitiveness relationship. *J. Econ. Perspect.* 9 97–118. 10.1257/jep.9.4.97

[B54] RasoolA.JundongH.SohailM. T. (2017). Relationship of intrinsic and extrinsic rewards on job motivation and job satisfaction of expatriates in China. *J. Appl. Sci.* 17 116–125. 10.3923/jas.2017.116.125

[B55] Sánchez-MedinaP. S.Díaz-PichardoR.Bautista-CruzA.Toledo-LópezA. (2015). Environmental compliance and economic and environmental performance: evidence from handicrafts small businesses in Mexico. *J. Bus. Ethics* 126 381–393. 10.1007/s10551-013-1945-2

[B56] SchalteggerS.SynnestvedtT. (2002). The link between ‘green’and economic success: environmental management as the crucial trigger between environmental and economic performance. *J. Environ. Manage.* 65 339–346. 10.1006/jema.2002.0555 12369398

[B57] ShahabA.ShihuaQ.RashidA.HasanF. U.SohailM. T. (2016). Evaluation of water quality for drinking and agricultural suitability in the lower indus plain in sindh province. Pakistan. *Polish J. Environ. Stud.* 25 2563–2574. 10.15244/pjoes/63777

[B58] SohailM. T.AftabR.MahfoozY.YasarA.YenY.ShaikhS. A. (2019a). Estimation of water quality, management and risk assessment in Khyber Pakhtunkhwa and Gilgit-Baltistan, Pakistan. *Desalination Water Treatment* 171:105. 10.5004/dwt.2019.24925 26354686

[B59] SohailM. T.MahfoozY.AzamK.YenY.GenfuL.FahadS. (2019b). Impacts of urbanization and land cover dynamics on underground water in Islamabad, Pakistan. *Desalin Water Treat* 159 402–411. 10.5004/dwt.2019.24156 26354686

[B60] SohailM. T.DelinH.SiddiqA. (2014a). Indus basin waters a main resource of water in Pakistan: an analytical approach. *Curr. World Environ.* 9:670. 10.12944/CWE.9.3.16

[B61] SohailM. T.DelinH.TalibM. A.XiaoqingX.AkhtarM. M. (2014b). An analysis of environmental law in Pakistan-policy and conditions of implementation. *Res. J. Appl. Sci. Eng. Technol.* 8 644–653. 10.19026/rjaset.8.1017

[B62] SohailM. T.EhsanM.RiazS.ElkaeedE. B.AwwadN. S.IbrahiumH. A. (2022a). Investigating the drinking water quality and associated health risks in metropolis area of Pakistan. *Front. Mater.* 9:864254. 10.3389/fmats.2022.864254

[B63] SohailM. T.ElkaeedE. B.IrfanM.Acevedo-DuqueÁMustafaS. (2022b). Determining Farmers’ awareness about climate change mitigation and wastewater irrigation: a pathway towards green and sustainable development. *Front. Environ. Sci.* 10:900193. 10.3389/fenvs.2022.900193

[B64] SohailM. T.MajeedM. T.ShaikhP. A.AndlibZ. (2022c). Environmental costs of political instability in Pakistan: policy options for clean energy consumption and environment. *Environ. Sci. Pollution Res.* 29 25184–25193. 10.1007/s11356-021-17646-5 34837622

[B65] SohailM. T.HuangD.BaileyE.AkhtarM. M.TalibM. A. (2013). Regulatory framework of mineral resources sector in Pakistan and investment proposal to Chinese companies in Pakistan. *Am. J. Industrial Bus. Manag.* 3:514. 10.4236/ajibm.2013.35059

[B66] SohailM. T.LinX.LizhiL.RizwanullahM.NasrullahM.XiuyuanY. (2021a). Farmers’ awareness about impacts of reusing wastewater, risk perception and adaptation to climate change in Faisalabad District, Pakistan. *Pol. J. Environ. Stud.* 30 4663–4675. 10.15244/pjoes/134292

[B67] SohailM. T.UllahS.MajeedM. T.UsmanA. (2021b). Pakistan management of green transportation and environmental pollution: a nonlinear ARDL analysis. *Environ. Sci. Pollution Res.* 28 29046–29055. 10.1007/s11356-021-12654-x 33548040PMC8222009

[B68] SohailM. T.UllahS.MajeedM. T.UsmanA.AndlibZ. (2021c). The shadow economy in South Asia: dynamic effects on clean energy consumption and environmental pollution. *Environ. Sci. Pollution Res.* 28 29265–29275. 10.1007/s11356-021-12690-7 33559075PMC8222016

[B69] SohailM. T.XiuyuanY.UsmanA.MajeedM. T.UllahS. (2021d). Renewable energy and non-renewable energy consumption: assessing the asymmetric role of monetary policy uncertainty in energy consumption. *Environ. Sci. Pollution Res.* 28 31575–31584. 10.1007/s11356-021-12867-0 33608782

[B70] SohailM. T.MahfoozbY.AftabcR.YendY.TalibeM. A.RasoolfA. (2020). Water quality and health risk of public drinking water sources: a study of filtration plants installed in Rawalpindi and Islamabad, Pakistan. *Desalination Water Treat* 181 239–250. 10.5004/dwt.2020.25119 26354686

[B71] SohailM. T.DelinH.SiddiqA.IdreesF.ArshadS. (2015). Evaluation of historic Indo-Pak relations, water resource issues and its impact on contemporary bilateral affairs. *Asia Pac. J. Multidiscip. Res.* 3 48–55.

[B72] UllahS.OzturkI.UsmanA.MajeedM. T.AkhtarP. (2020). On the asymmetric effects of premature deindustrialization on CO2 emissions: evidence from Pakistan. *Environ. Sci. Pollution Res.* 27 13692–13702. 10.1007/s11356-020-07931-0 32034591

[B73] UsmanA.OzturkI.HassanA.ZafarS. M.UllahS. (2021). The effect of ICT on energy consumption and economic growth in South Asian economies: an empirical analysis. *Telematics Inform.* 58:101537. 10.1016/j.tele.2020.101537

[B74] Van KampI.LeidelmeijerK.MarsmanG.De HollanderA. (2003). Urban environmental quality and human well-being: towards a conceptual framework and demarcation of concepts; a literature study. *Landscape Urban Plann.* 65 5–18. 10.1016/S0169-2046(02)00232-3

[B75] WeiX.RenH.UllahS.BozkurtC. (2022). Does environmental entrepreneurship play a role in sustainable green development? evidence from emerging Asian economies. *Econ. Res. Ekon. Istraživanja.* 1–13. 10.1080/1331677X.2022.2067887

[B76] YasaraA.FarooqaT.TabindaaA. B.SohailbM. T.MahfoozaY.MalikaA. (2019). Macrophytes as potential indicator of heavy metals in river water. *Desalination Water Treatment* 142 272–278. 10.5004/dwt.2019.23433 26354686

[B77] YatY. E. N.YuminS. H. I.SoeungB.SohailM. T. (2018). Victimization of the substance abuse and sexual behaviors among junior high school students in Cambodia. *Iran. J. Public Health* 47:357. 29845023PMC5971172

[B78] YenY.WangZ.ShiY.XuF.SoeungB.SohailM. T. (2017). The predictors of the behavioral intention to the use of urban green spaces: the perspectives of young residents in Phnom Penh. Cambodia. *Habitat Int.* 64 98–108. 10.1016/j.habitatint.2017.04.009

[B79] YenY.ZhaoP.SohailM. T. (2021). The morphology and circuity of walkable, bikeable, and drivable street networks in Phnom Penh, Cambodia. *Environ. Plann. B: Urban Anal. City Sci.* 48 169–185. 10.1177/2399808319857726

[B80] ZahidR. M. A.KhurshidM.KhanW. (2022). Do chief executives matter in corporate financial and social responsibility performance nexus? a dynamic model analysis of chinese firms. *Front. Psychol.* 13:897444. 10.3389/fpsyg.2022.897444 35712198PMC9197315

[B81] ZhangD.OzturkI.UllahS. (2022). Institutional factors-environmental quality nexus in BRICS: a strategic pillar of governmental performance. *Econ. Res. Ekon. Istraživanja.* 1–13. 10.1080/1331677X.2022.2037446

[B82] ZhaoP.YenY.BaileyE.SohailM. T. (2019). Analysis of urban drivable and walkable street networks of the ASEAN Smart Cities Network. *ISPRS Int. J. Geo-Inform.* 8:459. 10.3390/ijgi8100459

[B83] ZhaoW.ChangM.YuL.SohailM. T. (2022a). Health and human wellbeing in China: do environmental issues and social change matter? *Front. Psychol.* 13:860321. 10.3389/fpsyg.2022.860321 35664190PMC9157178

[B84] ZhaoW.HuangfuJ.YuL.LiG.ChangZ.SohailM. T. (2022b). Analysis on price game and supervision of natural gas pipeline tariff under the background of pipeline network separation in China. *Polish J. Environ. Stud.* 31 2961–2972. 10.15244/pjoes/145603

[B85] ZhenyuW.SohailM. T. (2022). Short-and long-run influence of education on subjective well-being: the role of ICT in China. *Front. Psychol.* 13:927562. 10.3389/fpsyg.2022.927562 35774959PMC9237439

[B86] ZhouG.LiH.OzturkI.UllahS. (2022). Shocks in agricultural productivity and CO2 emissions: new environmental challenges for China in the green economy. *Econ. Res. Ekon. Istraživanja.* 1–17. 10.1080/1331677X.2022.2037447

